# Mitochondrial Fission and Mitophagy Reciprocally Orchestrate Cardiac Fibroblasts Activation

This article has been retracted.

**DOI:** 10.3389/fcell.2020.629397

**Published:** 2021-01-21

**Authors:** Qing-Yuan Gao, Hai-Feng Zhang, Jun Tao, Zhi-Teng Chen, Chi-Yu Liu, Wen-Hao Liu, Mao-Xiong Wu, Wen-Yao Yin, Guang-Hao Gao, Yong Xie, Ying Yang, Pin-Ming Liu, Jing-Feng Wang, Yang-Xin Chen

**Affiliations:** ^1^Department of Cardiology, Sun Yat-sen Memorial Hospital, Sun Yat-sen University, Guangzhou, China; ^2^Laboratory of Cardiac Electrophysiology and Arrhythmia in Guangdong Province, Guangzhou, China; ^3^Department of Cardiovascular Surgery, Sun Yat-sen Memorial Hospital, Sun Yat-sen University, Guangzhou, China

**Keywords:** cardiac fibroblasts, mitochondrial fission, glycolysis, reactive oxygen species, mitophagy

## Abstract

Although mitochondrial fission has been reported to increase proliferative capacity and collagen production, it can also contribute to mitochondrial impairment, which is detrimental to cell survival. The aim of the present study was to investigate the role of mitochondrial fission in cardiac fibroblasts (CF) activation and explore the mechanisms involved in the maintenance of mitochondrial health under this condition. For this, changes in the levels of mitochondrial fission/fusion-related proteins were assessed in transforming growth factor beta 1 (TGF-β1)-activated CF, whereas the role of mitochondrial fission during this process was also elucidated, as were the underlying mechanisms. The interaction between mitochondrial fission and mitophagy, the main defense mechanism against mitochondrial impairment, was also explored. The results showed that the mitochondria in TGF-β1-treated CF were noticeably more fragmented than those of controls. The expression of several mitochondrial fission-related proteins was markedly upregulated, and the levels of fusion-related proteins were also altered, but to a lesser extent. Inhibiting mitochondrial fission resulted in a marked attenuation of TGF-β1-induced CF activation. The TGF-β1-induced increase in glycolysis was greatly suppressed in the presence of a mitochondrial inhibitor, whereas a glycolysis-specific antagonist exerted little additional antifibrotic effects. TGF-β1 treatment increased cellular levels of reactive oxygen species (ROS) and triggered mitophagy, but this effect was reversed following the application of ROS scavengers. For the signals mediating mitophagy, the expression of Pink1, but not Bnip3l/Nix or Fundc1, exhibited the most significant changes, which could be counteracted by treatment with a mitochondrial fission inhibitor. Pink1 knockdown suppressed CF activation and mitochondrial fission, which was accompanied by increased CF apoptosis. In conclusion, mitochondrial fission resulted in increased glycolysis and played a crucial role in CF activation. Moreover, mitochondrial fission promoted reactive oxygen species (ROS) production, leading to mitophagy and the consequent degradation of the impaired mitochondria, thus promoting CF survival and maintaining their activation.

## Introduction

Cardiac fibroblasts (CF) play a critical role in maintaining the normal structure and proper function of the heart and are also a determinant cell type in cardiac remodeling. CF are activated and deposit extracellular matrix (ECM) proteins following injury, thereby helping to repair and remodel the heart. However, studies have also shown that CF are the main cellular effectors of heart failure through the deposition of stiff ECM in the cardiac interstitium (Humeres and Frangogiannis, 2019), which results in reduced cardiac output and ventricular compliance and leads to poor prognosis.

Under normal conditions, CF activation refers to the transition of the hemostatic phenotype and exhibits remarkable phenotypic plasticity. These CF transform to myofibroblasts; fibrotic proteins are dramatically increased; and the capacity of proliferation, migration, and matrix deposition is significantly enhanced. Several mechanisms have been proposed to explain how CF are activated, among which metabolic reprogramming is thought to be critical. For instance, we recently demonstrated that enhanced glycolysis is crucial for CF activation (Chen et al., 2020b). Glycolysis and mitochondrial respiration are the major energy-yielding manners. They are highly interacted, and mitochondrial alteration is a vital regulator of glycolysis (Bertram et al., 2007). Mitochondrial dynamics are widely accepted as being important regulators of glycolytic flux. Enhanced mitochondrial fission or defective fusion results in the fragmented mitochondria and increased glycolysis (Hagenbuchner et al., 2013; Rossin et al., 2015).

Increased mitochondrial fission is associated with right ventricular fibroblasts proliferation and collagen production (Tian et al., 2018). However, whether mitochondrial fission plays a role in CF activation remains unknown. Moreover, mitochondrial fission usually generates the impaired mitochondria, leads to excessive mitochondrial reactive oxygen species (mtROS) production, and induces apoptosis, which greatly challenges its prosurvival effects (Bras et al., 2007; Vantaggiato et al., 2019; Wang et al., 2020a). Consequently, an understanding of the detailed role of mitochondrial fission during CF activation merits further investigation.

It seems plausible that there may be a mechanism that mitigates the harmful effects of mitochondrial fission and helps maintain mitochondrial health. Mitophagy, which is primarily triggered by elevated mtROS levels, is the main safeguard mechanism against disrupted mitochondrial homeostasis (Frank et al., 2012; Ajoolabady et al., 2020; Schofield and Schafer, 2020; Wang et al., 2020d). Mitophagy is a selective autophagic process for the removal of the damaged mitochondria and is vital for cell survival. Mitophagy has been reported to be activated by profibrotic stimuli and to play a key role in fibroblasts activation and organ fibrosis (Li et al., 2020). Consequently, the aim of the current study was to investigate the role of mitochondrial fission in CF activation. The interaction between mitochondrial fission and mitophagy during this process is also detailed.

## Materials and Methods

### Cell Culture, Treatment, and Small Interfering RNA Transfection

Neonatal mouse CF (NMCF) were prepared from the hearts of 1–3-day-old C57BL/6 mice (Takeda et al., 2010). Briefly, heart ventricles were separated, digested, and gently shaken in D-Hanks Balanced Salt Solution (Sigma-Aldrich, Saint Louis, MO, USA) with 0.2% type 2 collagenase (Gibco, Carlsbad, CA, USA) in an incubator at 37°C. The digested suspensions were plated on culture dishes with Dulbecco's Modified Eagle's Medium/Ham's F-12 Nutrient Mixture (DMEM/F12; Gibco) supplemented with 10% fetal bovine serum (FBS; Gibco) for 90 min at 37°C in humidified air with 5% CO_2_. After washing, the attached NMCF were cultured in DMEM/F12. Experiments were carried out after one passage, and the cells were kept in DMEM/F12 containing 1% FBS for 12 h before treatment. Cultured NMCF were treated with 5 ng/ml transforming growth factor beta 1 (TGF-β1; R&D Systems, Minneapolis, MN, USA) in the presence or absence of mitochondrial division inhibitor 1 (mdivi-1, 5 μM; Sigma-Aldrich), 2-deoxy-d-glucose (2-DG, 1 mM; Sigma-Aldrich), N-acetylcysteine (NAC, 5 mM; Sigma-Aldrich), or MitoTEMPO (5 μM; Sigma-Aldrich).

For small interfering RNA (siRNA) transfection, siRNA [against the target gene or nonsense control (NC)] was transfected into NMCF at a concentration of 50 nM using Lipofectamine RNAiMAX (Invitrogen, Carlsbad, CA, USA) 24 h before treatment [TGF-β1 or phosphate-buffered saline (PBS)]. Two siRNA oligonucleotides targeting one gene were used to avoid off-target effects. All siRNAs were obtained from RiboBio (Guangzhou, Guangdong, China). The siRNA sequences are listed in Supplementary Table 1.

### Analysis of Mitochondrial Morphology in CF

Treated NMCF (1 × 10^5^) were stained with 200 μM MitoTracker Deep Red (Thermo Fisher Scientific, Carlsbad, CA, USA) at 37°C for 30 min. Images were captured using a laser scanning confocal microscope (Zeiss LSM800, Germany). For analyses, the volume and the mean (area/perimeter)/circularity index of the mitochondrial network was calculated using the Mito-Morphology macro in ImageJ (NIH, Bethesda, MD, USA) (Simula et al., 2018).

### Transmission Electron Microscopic Analyses

For transmission electron microscopic (TEM) observation, NMCF (1 × 10^7^) were harvested by scraping and fixed in 2.5% glutaraldehyde/0.1 M sodium cacodylate buffer (pH 7.2) for 1 h, followed by a 2-h incubation in 1% osmium tetroxide at the same pH. The samples were then stained, dehydrated, embedded, cut into ultrathin sections (70 nM), and contrasted with 1.2% uranyl acetate and lead citrate. Images were acquired with an HT7800 TEM (Hitachi, Tokyo, Japan) at 80 kV. ImageJ software was used for mitochondrial area analyses.

### Isolation of the Mitochondria

After treatment, the mitochondria were fractionated using a mitochondrial isolation kit for cultured cells (1 × 10^7^) (Thermo Fisher Scientific) according to the manufacturer's instructions. To ensure the purity of the fraction, COXIV and GAPDH were respectively used as mitochondrial and cytosolic markers.

### Measurements of the Oxygen Consumption Rate and Extracellular Acidification Rate

The oxygen consumption rate (OCR) was measured using a Seahorse XF Cell Mito Stress Test Kit (Agilent, DE, USA), and the extracellular acidification rate (ECAR) was detected using a Seahorse XF Glycolytic Rate Assay Kit (Agilent) in an Agilent Seahorse Extracellular Flux Analyzer (Agilent). Briefly, the cells (2 × 10^4^) were seeded in Seahorse cell culture microplates and incubated at 37°C overnight. The cultured medium was changed to XF assay medium, and the plates were placed in an incubator at 37°C without CO_2_ for 1 h. The OCR was measured by the sequential injections of 1 μM oligomycin, 1 μM carbonyl cyanide 4-(trifluoromethoxy)phenylhydrazone (FCCP), and 1 μM rotenone plus antimycin A (mitochondrial stress test). The ECAR was measured by the sequential injection of 0.5 μM rotenone plus antimycin A and 50 mM 2-DG (glycolytic rate assay).

### Assessment of mtROS Production

mtROS were detected in NMCF (1 × 10^5^) by staining with 10 μM MitoSOX Red (Invitrogen) at 37°C for 10 min. After staining, the cells were washed and then either imaged with a confocal microscope (Zeiss LSM800) or analyzed by flow cytometry; in the latter case, fluorescence signals were detected at 580 nm.

### Cell Proliferation Assay

NMCF proliferation was measured using the CellTiter 96® AQueous One Solution Cell Proliferation Assay Kit (Promega, Fitchburg, WI, USA) and the Cell-Light™ EdU Apollo 567 *in vitro* kit (RiboBio) according to the manufacturer's instructions. In brief, 20 μl of CellTiter 96 AQueous One Solution, containing 3-(4,5-dimethylthiazol-2-yl)-5-(3-carboxymethoxyphenyl)-2-(4-sulfophenyl)-2H-tetrazolium (MTS), was added to each well (containing 1 × 10^4^ CF in 100 μl of medium), and absorbance at 490 nm was recorded 1 h later. For EdU detection, fixed cells (1 × 10^4^) were stained with Apollo 567 according to the manufacturer's instructions. Images were captured under a fluorescence microscope. The cell proliferation rate was assessed as the proportion of EdU-positive cells.

### Wound Healing Assay

A wound was made in a continuous monolayer of NMCF (2 × 10^5^) by scratching a line across the bottom of the well with a sterile pipette tip. The cellular debris was washed off with PBS, and the cells were cultured with different treatments. Images were taken in the same scratch area at 0 and 24 h. The proportion of migrated cells was calculated using ImageJ software.

### Cell Apoptosis Assay

The cell apoptosis assay was performed with the FITC Annexin V/Dead Cell Apoptosis Kit (Invitrogen) following the manufacturer's instructions and as previously described (Mai et al., 2018). Briefly, after the respective treatments, 2 × 10^5^ cells were harvested and resuspended in annexin-binding buffer, followed by sequential incubation with annexin V (15 min) and propidium iodide. Fluorescence signals were detected at 518 and 617 nm for FITC and propidium iodide, respectively.

### Gelatin Zymography Assay

The activity of matrix metalloproteinase (MMP)-2 and MMP-9 in CF was measured using a gelatin zymography kit (Cosmo Biological Corporation, Tokyo, Japan) according to the manufacturer's instructions. In brief, 30 μg of each sample was loaded for electrophoresis, washed, and incubated at 37°C. After Coomassie blue staining, the gels were scanned, and ImageJ was used for densitometric analysis.

### Lysyl Oxidase Activity Assay

Lysyl oxidase (LOX) activity was measured using the Lysyl Oxidase Activity Assay Kit (Abcam, Cambridge, UK) following the manufacturer's instructions. Briefly, cell culture supernatants were collected and incubated for 30 min in the presence of 50 μl of the reaction mixture. Fluorescence was monitored with a fluorescence plate reader at 540/590 nm excitation/emission wavelengths.

### Immunofluorescence and Colocalization Analysis of Drp1 and Tomm20

The cells were washed three times with PBS and fixed in 4% paraformaldehyde (Sigma-Aldrich) for 30 min, permeabilized with 0.5% Triton X-100 (Sigma-Aldrich) for 20 min, and then blocked with 5% bovine serum albumin (BSA; Sigma-Aldrich) for 1 h at room temperature. The cells were incubated at 4°C overnight with primary antibodies against Drp1 (NB110-55288, 1:100; Novus Biologicals, Minneapolis, MN, USA), Tomm20 (sc-17764, 1:50; Santa Cruz Biotechnology, Santa Cruz, CA, USA), α-SMA (ab7817, 1:200; Abcam), and vimentin (5741S, 1:200; Cell Signaling Technology, Danvers, MA, USA). The next day, the cells were incubated with the appropriate secondary antibodies [Alexa Fluor 488-conjugated anti-rabbit IgG (ab150077, 1:500; Abcam) for Drp1 and vimentin and Alexa Fluor 594-conjugated anti-mouse IgG (ab150116, 1:500; Abcam) for Tomm20 and α-SMA] for 1 h at room temperature in the dark. Nuclei were counterstained with DAPI (62242, 1:1,000; Thermo Fisher Scientific). Samples were analyzed by either fluorescence or confocal microscopy. To determine immunofluorescence intensity, the signals were converted to average grayscale intensity and subsequently analyzed using ImageJ. The Coloc 2 plugin in ImageJ was used to analyze colocalization between Drp1 and Tomm20.

### Immunoblotting Analyses

Protein levels were measured by immunoblotting. In brief, total proteins were extracted using a protein extraction kit (Cell Signaling Technology). The proteins were then separated by SDS-PAGE, transferred to polyvinylidene difluoride (PVDF) membranes (Millipore, Bedford, MA, USA), blocked in 5% BSA, and incubated with primary antibodies targeting the following proteins: Drp1 (NB110-55288, 1:1,000; Novus Biologicals), p-Drp1^Ser616^ (PA5-64821, 1:1,000; Invitrogen), Fis1 (NB100-56646, 1:1,000; Novus Biologicals), Mff (84580S, 1:1,000; Cell Signaling Technology), Mfn2 (9482S, 1:1,000; Cell Signaling Technology), Opa1 (67589S, 1:1,000; Cell Signaling Technology), β-actin (4970S, 1:1,000; Cell Signaling Technology), COXIV (4844S, 1:1,000; Cell Signaling Technology), GAPDH (5174S, 1:1,000; Cell Signaling Technology), Col1a1 (ab21286, 1:1,000; Abcam), Ctgf (MAB91901, 1:500; R&D Technology), Tsp1 (37879S, 1:1,000; Cell Signaling Technology), Postn (NBP1-82472, 1:1,000; Novus Biologicals), S100A4 (AF4138, 1:1,000; Novus Biologicals), Sparc (8725S, 1:1,000; Cell Signaling Technology), Pfkfb3 (13123S, 1:1,000; Cell Signaling Technology), Pdh (3205S, 1:1,000; Cell Signaling Technology), Pink1 (BC100-494, 1:1,000; Novus Biologicals), Parkin (4211S, 1:1,000; Cell Signaling Technology), Bnip3l/Nix (12396S, 1:1,000; Cell Signaling Technology), and Fundc1 (ab224722, 1:1,000; Abcam). The secondary antibodies used were HRP-conjugated anti-rabbit IgG (7074S, 1:2,000; Cell Signaling Technology), anti-mouse IgG (7076S, 1:2,000; Cell Signaling Technology), and anti-sheep IgG (HAF016, 1:1,000; R&D Technology). Enhanced electrochemiluminescence (Millipore, Billerica, MA, USA) was used to visualize the protein bands. ImageJ was used for densitometric measurements of the bands.

### Statistical Analyses

Data were presented as mean ± standard error of the mean (SEM). One-way ANOVA was used to analyze differences among multiple groups, followed by the Student–Newman–Keuls (SNK) *post- hoc* test. The two-tailed Student's *t*-test was used for comparisons between two groups. Statistical analysis was carried out using R v3.6.1. A *P*-value < 0.05 was considered significant.

## Results

### Mitochondrial Fission Was Increased During CF Activation

To observe changes in the mitochondria during CF activation, we directly visualized mitochondrial morphology following TGF-β1 treatment using MitoTracker Deep Red staining. The results showed that the mitochondria in CF were more fragmented than controls; however, this effect could be reversed by the application of mdivi-1 (Figure 1A). Besides, the smaller mitochondria induced by TGF-β1 were also observed in the TEM analysis (Figure 1B).

**Figure 1:** Mitochondrial fission was increased during CF activation. **(A)** MitoTracker Deep Red staining was used to observe the mitochondrial morphology of cardiac fibroblasts (CF). Mitochondrial volume and the mean (area/perimeter)/circularity index was calculated using ImageJ. **(B)** Transmission electron microscopy (TEM) was employed to directly observe the fragmented mitochondria. Mitochondrial area and length were also measured using ImageJ. **(C)** The expression of fission-related and fusion-related proteins following TGF-β1 plus mdivi-1 cotreatment was measured in whole-cell lysates *via* immunoblotting. **(D)** Immunoblotting, with quantification, of the same proteins in mitochondrial and cytoplasmic fractions. COXIV was used as the loading control for mitochondrial proteins. **(E)** The translocation of Drp1 to the mitochondrial membrane was observed by confocal microscopy. Colocalization was analyzed using the Coloc 2 plugin in ImageJ. Data are shown as mean ± standard error of the mean (*n* = 3 independent cell isolations per group). Means were compared using one-way ANOVA, followed by the Student–Newman–Keuls (SNK) *post hoc* test. *P < 0.05; **P < 0.01; ***P < 0.001.

Because mitochondrial fission and fusion are the main mechanisms regulating mitochondrial morphology, we examined the changes in the levels of key proteins associated with mitochondrial fission and fusion. Whole-cell lysate analysis showed that the levels of all the mitochondrial fission-related proteins–total Drp1, p-Drp1^Ser616^, Mff, and Fis1–were significantly upregulated by TGF-β1 treatment (Figure 1C), whereas the levels of the mitochondrial fusion-related proteins–Mfn2 and Opa1–showed a slight decrease (Figure 1C); as observed for mitochondrial morphology, these effects could also be rescued by treatment with mdivi-1. Similar results were recorded for mitochondrial proteins (Figure 1D). Confocal microscopic analysis of Drp1 and Tomm20 (a mitochondrial membrane marker) showed that TGF-β1 treatment increased the levels of Drp1 in both the mitochondria and the cytoplasm (Figure 1E). Combined, these results demonstrated that TGF-β1 treatment independently and markedly increased the incidence of mitochondrial fission.

### Inhibition of TGF-β1-Induced Mitochondrial Fission Abolished CF Activation

We further explored the role of mitochondrial fission during TGF-β1-dependent CF activation. As shown in Figures 2A,B, the inhibition of mitochondrial fission attenuated the expression of various CF activation markers (α-SMA, Postn, and Ctgf). Regarding cell proliferation, TGF-β1 treatment resulted in increased and stronger EdU staining (Figure 2C) and increased MTS assay values (Figure 2D); however, both were greatly suppressed with the coadministration of mdivi-1. Immunological staining of vimentin, a mesenchymal cell marker, also revealed a moderate decrease in the number of vimentin-positive cells with TGF-β1 and mdivi-1 cotreatments (Figure 2C).

**Figure 2:** The inhibition of TGF-β1-induced mitochondrial fission abolished cardiac fibroblasts (CF) activation. **(A)** α-SMA immunofluorescence staining and semi-quantitative analysis. **(B)** The expression of the markers of CF activation, Postn and Ctgf, was measured by immunoblotting. EdU and vimentin staining **(C)** and an MTS assay **(D)** were used to observe CF proliferation**. (E)** Gelatin zymography was used to measure MMP-2 and MMP-9 activities. **(F)** The activity of lysyl oxidase (LOX) was used as an indicator of extracellular matrix (ECM) deposition. **(G)** Immunoblot of ECM-related proteins, with quantification, following TGF-β1 plus mdivi-1 cotreatment. **(H)** A wound healing assay was employed to evaluate CF migration. Data are shown as mean ± standard error of the mean (*n* = 3 independent cell isolations per group). Means were compared using one-way ANOVA, followed by the Student–Newman–Keuls (SNK) *post hoc* test. *P < 0.05; **P < 0.01; ***P < 0.001.

In addition to suppressing proliferation, the inhibition of mitochondrial fission also suppressed ECM deposition and CF migration. Mdivi-1 treatment abolished the activity of MMP-2 and MMP-9 (Figure 2E) and decreased various ECM deposition-related proteins, including LOX activity and expressions of Col1a1, Tsp1, S100A4, and Sparc (Figures 2F,G). A wound healing assay indicated that inhibiting mitochondrial fission also reduced CF migration (Figure 2H). Together, these results demonstrated that the inhibition of TGF-β1-induced mitochondrial fission significantly suppressed CF activation.

### Reduced CF Glycolytic Flux Could Be Important for the Mitochondrial Fission Inhibition-Induced Suppression of CF Activation

The above results clearly showed a causality between TGF-β1-induced mitochondrial fission and CF activation. However, the mechanisms underlying the antifibrotic effects conferred by treatment with the mitochondrial fission inhibitor mdivi-1 remained unknown. Based on our previous report demonstrating the crucial role of glycolysis during CF activation and the close relationship between mitochondrial fission and glycolysis, we investigated how mdivi-1 treatment would affect glycolysis in CF.

As expected, mdivi-1 treatment decreased glycolytic flux, as indicated by the observed decrease in the ECAR and the increase in the OCR (Figures 3A,B). Meanwhile, compared with TGF-β1 treatment alone, the expression of the key glycolytic enzymes, Pfkfb3 and Pdh, was significantly suppressed by cotreatment with mdivi-1 (Figure 3C). Moreover, we found that, in the presence of the mitochondrial fission inhibitor, the antifibrotic effects of the glycolysis inhibitor, 2-DG, were almost abolished (Figure 3D). These data implied that the inhibition of glycolysis could be the key mechanism underlying the antifibrotic effects of mitochondria fission inhibition.

**Figure 3:** Reducing the cardiac fibroblasts (CF) glycolytic flux may be important for mitochondrial fission inhibition-induced suppression of CF activation. **(A)** Measurements of the extracellular acidification rate (ECAR) metabolic profile by Seahorse XF glycolytic rate assay kit and analyses of CF Proton Efflux Rate (PER) in basal glycolysis and glycolysis capacity. **(B)** The oxygen consumption rate (OCR) as measured using a Seahorse XF Cell Mito Stress Test Kit and analyses of the OCR under basal and maximum respiration. **(C)** Western blot analyses and quantification of key glycolytic enzymes under TGF-β1 plus mdivi-1 cotreatment. **(D)** The expression of CF activation-related markers was measured by immunoblotting following TGF-β1 plus mdivi-1 cotreatment and in the presence or absence of 2-DG. Data are shown as mean ± standard error of the mean (*n* = 3 independent cell isolations per group). Means were compared by one-way ANOVA, followed by the Student–Newman–Keuls (SNK) *post hoc* test. ns, not significant; *P < 0.05; **P < 0.01; ***P < 0.001.

### mtROS Was the Key Instigator of Mitophagy in CF

The process of mitochondrial fission is known to generate the impaired mitochondria, which may be detrimental to the cells. However, the above data clearly showed that mitochondrial fission promoted CF activation, proliferation, migration, and ECM deposition without exerting detrimental effects.

Therefore, we first investigated mtROS generation. As determined by both flow cytometry and confocal microscopy, MitoSOX staining indicated that mtROS production was significantly increased in TGF-β1-treated CF, an effect that was also markedly attenuated with mdivi-1 application (Figures 4A,B). Subsequently, we sought to determine the mechanisms involved in safeguarding against the detrimental effects associated with the impaired mitochondria. Because excessive mtROS production is thought to be the main endogenous trigger for mitophagy, we next made use of ROS scavengers to assess the causality between increased mtROS generation and the incidence of mitophagy. We first treated CF with TGF-β1 and tested the three canonical pathways that are known to activate mitophagy. We found that the expression of Pink1 was substantially increased, whereas that of Fundc1 and Bnip3l/Nix was scarcely changed (Figure 4C). Similar changes were also found for the expression of mitochondrial fractions. Importantly, we found that Parkin was also recruited to the mitochondria in the presence of TGF-β1 (Figure 4D). These data suggested that TGF-β1 induced mitophagy through the activation of the Pink1/Parkin signal. Moreover, as shown in Figures 4C,D, the application of the ROS scavengers NAC and mito-Tempo significantly suppressed the expression of Pink1 in both whole-cell and mitochondrial extracts and abolished Parkin recruitment to the mitochondria.

**Figure 4:** Mitochondrial reactive oxygen species (mtROS) were the main instigators of mitophagy in cardiac fibroblasts (CF). mtROS was detected by MitoSOX staining and visualized by flow cytometry **(A)** and confocal microscopy. **(B)** Mean immunofluorescence intensities were calculated. **(C)** The expression of mitophagy-related proteins after treatment with TGF-β1 and ROS scavengers was measured in whole-cell lysates. **(D)** Western blotting was used to compare mitophagy-related parameters and mitochondrial parkin translocation in particular, among the different groups. COXIV was used as the loading control for the mitochondrial fraction. Data are shown as mean ± standard error of the mean (*n* = 3 independent cell isolations per group). Means were compared by one-way ANOVA, followed by the Student–Newman–Keuls (SNK) *post hoc*. ns, not significant; ***P < 0.001.

### Mitochondrial Fission Triggered Mitophagy in CF

Because we found that enhanced mitochondrial fission was accompanied by increased mtROS production, we next assessed the intrinsic interaction between mitochondrial fission and mitophagy. We further validated the incidence of mitophagy in CF under TGF-β1 treatment. TEM analysis revealed a mitochondrion enclosed in a double-membrane structure in TGF-β1-treated CF (Figure 5A). However, the mitophagosomes were rarely observed in the presence of the mitochondrial fission inhibitor mdivi-1 (Figure 5A). Furthermore, treatment with mdivi-1 almost completely blocked the increase in Pink1 expression (Figure 5B), and similar changes regarding Pink1 were found in mitochondrial proteins (Figure 5C). Importantly, Parkin recruitment to the mitochondria was also abolished by treatment with the mitochondrial fission inhibitor (Figure 5C). These findings showed that TGF-β1-induced mitochondrial fission triggered mitophagy in activated CF.

**Figure 5:** Mitochondrial fission triggered mitophagy in cardiac fibroblasts (CF). **(A)** Transmission electron microscopy (TEM) was used to observe the mitophagosomes in TGF-β1-treated CF exposed or not to a mitochondrial fission inhibitor. The black arrows indicate the mitophagosomes in CF. The number of the mitochondria and the mitophagosomes was calculated. **(B)** Immunoblotting and quantification of mitophagy-related proteins from whole-cell lysates derived from CF treated or not with mdivi-1 and exposed to TGF-β1. **(C)** The expression of mitophagy-related proteins and parkin mitochondrial translocation in mitochondrial and cytoplasmic fractions of the indicated groups were assessed by immunoblotting. COXIV was used as the loading control for mitochondrial proteins. Data are shown as mean ± standard error of the mean (*n* = 3 independent cell isolations per group). Means were compared by one-way ANOVA, followed by the Student–Newman–Keuls (SNK) *post hoc* test. *P < 0.05; ***P < 0.001.

### Mitophagy Inhibition Suppressed Mitochondrial Fission and CF Activation

The above results indicated that mtROS generated through mitochondrial fission triggered mitophagy, which could serve as a safeguard mechanism and was important for attenuating the detrimental effects resulting from mitochondrial fission. However, the effects of mitophagy on mitochondrial fission and CF activation were still unknown. We, therefore, continued to explore the effects of mitophagy on mitochondrial fission and CF activation.

As shown by MitoTracker Deep Red staining (red fluorescence) in Figure 6A, treatment with Pink1 siRNA resulted in more continuous mitochondria than the mitochondrial fragmentation resulting from TGF-β1 application. In addition, the expression of Drp1 and Mff, markers of mitochondrial dynamics, was substantially decreased in CF transfected with Pink1 siRNA treatment. Notably, however, p-Drp1^ser616^ was suppressed to a much greater extent than Drp1 and Mff (Figure 6B). In contrast, Mfn2 levels were also significantly increased by Pink1 siRNA treatment, whereas the expression of Opa1 was only marginally changed (Figure 6B).

**Figure 6:** Inhibiting mitophagy suppressed mitochondrial fission. **(A)** MitoTracker Deep Red staining in cardiac fibroblasts (CF) transfected with either Pink1 siRNA or negative control (NC) and exposed to TGF-β1. **(B)** Immunoblotting analysis, with quantification, of mitochondrial fission- and fusion-related proteins among the different groups. Data are shown as mean ± standard error of the mean (*n* = 3 independent cell isolations per group). Means were compared by one-way ANOVA, followed by the Student–Newman–Keuls (SNK) *post hoc* test. *P < 0.05; **P < 0.01; ***P < 0.001.

Regarding CF activation, we found that Pink1 siRNA treatment suppressed the levels of CF markers (α-SMA immunofluorescence staining, Figure 7A; Postn and Ctgf expression, Figure 7B), as well as the proliferation (EdU and vimentin staining and MTS measurement, Figures 7C,D), migration (wound healing assay, Figure 7E), and ECM deposition (LOX activity, Figure 7F; Col1a1, Tsp1, Sparc, and S100A4 expression, Figure 7G) of CF. In addition, CF transfected with Pink1 siRNA underwent higher levels of apoptosis as detected by flow cytometry (Figure 7H), indicative of the crucial role of Pink1-induced mitophagy in maintaining cell health. Combined, these data demonstrated that suppressing mitophagy *via* Pink1 siRNA treatment inhibited mitochondrial fission and CF activation while inducing higher rates of CF apoptosis.

**Figure 7:** The suppression of mitophagy inhibited cardiac fibroblasts (CF) activation. CF were transfected with either Pink1 siRNA or negative control (NC) and then stimulated with TGF-β1. **(A)** α-SMA immunofluorescence staining and semi-quantitative analysis**. (B)** Immunoblot analyses and quantitative analyses of the markers of CF activation, Postn and Ctgf, among the different groups. EdU and vimentin staining **(C)** and the MTS cell proliferation assay **(D)** were used to evaluate CF proliferation. **(E)** A wound healing assay was performed to evaluate CF migratory capacity following the different treatments. **(F)** Measurement of lysyl oxidase (LOX) activity. (**G**) The relative expression levels of extracellular matrix (ECM)-related proteins normalized to that of beta-actin**. (H)** Cell apoptosis was compared among the different groups by flow cytometry. Data are shown as mean ± standard error of the mean (*n* = 3 independent cell isolations per group). Means were compared by one-way ANOVA, followed by the Student–Newman–Keuls (SNK) *post hoc* test. *P < 0.05; **P < 0.01; ***P < 0.001.

## Discussion

In the present study, we demonstrated that CF activation was accompanied by increased mitochondrial fission. Specifically, pharmacological inhibition of mitochondrial fission could effectively alleviate CF activation *in vitro*, which also mitigated the concomitant TGF-β1-induced mtROS release and metabolic switch in activated CF. Meanwhile, increased mitochondrial fission and mtROS generation triggered mitophagy, which further protected CF health and promoted CF activation and apoptosis resistance. The feed-forward mechanism between mitochondrial fission and mitophagy sustained CF activation and homeostasis.

The mechanisms orchestrating mitochondrial dynamics, including mitochondrial fission and fusion, are crucial for cell life and cellular energy metabolism through regulating mitochondrial morphology and functions. However, dysregulated mitochondrial dynamics, including enhanced mitochondrial fission, can lead to the reprogramming of energy metabolism, mitochondrial damage, and even disease (Westermann, 2010; Youle and van der Bliek, 2012; Willems et al., 2015). These effects have been implicated in organ fibrosis and associated with different types of fibroblasts, and the connection between mitochondrial fission and fibrotic events is further supported by both *in vitro* and *in vivo* evidence (Zhang et al., 2015, 2020; Tian et al., 2018; Tseng et al., 2019; Chen et al., 2020a; Wang et al., 2020e).

Studies have shown that mitochondrial fission can aggravate kidney, liver, and lung fibrogenesis (Zhang et al., 2015, 2020; Wang et al., 2020e). Furthermore, the suppression of mitochondrial fission not only can alleviate the activation and proliferation of renal fibroblasts but also can enhance apoptosis in both pulmonary and skin fibroblast. Referring to cultured CF, the inhibition of mitochondrial fission by mdivi-1 has been demonstrated to reduce collagen production (Tian et al., 2018; Tseng et al., 2019) and proliferation (Tian et al., 2018) in lysophosphatidylcholine-treated human CF and monocrotaline-induced right ventricular fibroblasts. However, these two models were not classical profibrotic CF models. Mitochondrial fission was also shown to play a progressive role in obesity-induced cardiac fibrosis in obese minipigs (Chen et al., 2020a); as with the above-mentioned studies, the authors used the H9C2 cardiomyocyte line and not CF as the *in vitro* model, which could not recapitulate the importance of mitochondrial fission in CF. According to our findings, mdivi-1 could reduce TGF-β1-induced mitochondrial fission, as well as activation, proliferation, collagen deposition, and migration of cultured CF, which was consistent with the conclusions of the aforementioned studies.

Taken together, our data highlighted the importance of mitochondrial fission as a driver of TGF-β1-induced CF activation. In addition, we also showed that mitochondrial fission exerted a detrimental influence on energy metabolism and mitochondrial homeostasis. However, our data indicated that a metabolic shift to glycolysis and evoked mitophagy may be the key mediators of the safeguard mechanisms that maintain cell health in parallel with CF activation.

Energy metabolism, and primarily oxidative phosphorylation (OXPHOS) and glycolysis, is vital for cell survival and function. Owing to the high energy demand of myofibroblasts (Li et al., 2016; Marín-Hernández et al., 2019), metabolic reprogramming and enhanced glycolysis are considered to be the drivers of fibroblast activation (Xie et al., 2015; Zhao et al., 2020). We previously obtained similar results, namely, that suppression of glycolysis can attenuate CF activation (Chen et al., 2020b). In contrast, unbalanced mitochondrial dynamics can disrupt mitochondrial energy supply. Enhanced mitochondrial fission was shown to induce metabolic reprogramming and a shift to glycolysis. Seo et al. suggested that knockout of mitochondrial fission-related genes in the embryonic stem cells, such as Drp1 and Mff, can increase OXPHOS and reduce glycolysis as a result of reduced mitochondrial fission (Seo et al., 2020). In addition, increasing mitochondrial fission by overexpressing Fis1 also induced glycolysis in an insulinoma cell line (Park et al., 2008). Specific to fibroblasts, because of excessive mitochondrial fission in renal- and cancer-associated myofibroblasts, the energy metabolism pattern switched from OXPHOS to glycolysis (Guido et al., 2012; Wang et al., 2020e). Nevertheless, to date, no study has conclusively explained how mitochondrial fission induces glycolysis, and further studies using genetic approaches are needed to identify the relevant mechanisms.

In addition to a switch to glycolysis, mitochondrial fission was also accompanied by mitochondrial impairment in parallel with increased mtROS production. Our findings revealed that mtROS levels were increased in TGF-β1-induced CF, which could nonetheless be reversed by the application of the mitochondrial fission inhibitor mdivi-1. This suggested that enhanced mitochondrial fission in activated CF was responsible for mtROS generation. Mitochondrial fission has been reported to contribute to mitochondrial impairment in other cell types, effects that could be rescued by inhibiting mitochondrial fission through the silencing of Drp1(Bras et al., 2007; Vantaggiato et al., 2019; Wang et al., 2020a). Mitochondrial fission/mtROS interaction can result in a positive feedback mechanism that can aggravate mitochondrial impairment, thereby hinting at the crucial role of mtROS generation in the detrimental effects associated with mitochondrial fission (Zhao et al., 2017). However, excessive mitochondrial fission and mtROS production can result in apoptosis in different cell types (Bras et al., 2007; Catanzaro et al., 2019; Vantaggiato et al., 2019; Zhou et al., 2019). In particular, after ischemia–reperfusion injury, treatment targeting the impaired mitochondria helped to protect against cell apoptosis and organ damage (Wang et al., 2020b,c; Zhou et al., 2020). Therefore, under the circumstances, it needed effective safeguard mechanisms against the impaired mitochondria, and mitophagy was essential for defending mitochondrial health and apoptosis resistance (Rana et al., 2017; Catanzaro et al., 2019; Zhou et al., 2019).

Mitophagy is thought to aid in the maintenance of cell homeostasis and may play an essential role in repairing mitochondrial fission-induced mitochondrial alterations. However, it is not clear whether mitophagy itself can regulate the process of mitochondrial fission. In the present study, we demonstrated that enhanced mitochondrial fission activated mitochondrial quality control mechanisms *via* increasing mtROS production. In turn, we also verified that mitophagy, an important component of the mitochondrial quality control system, could promote mitochondrial fission. This finding was consistent with previous studies that showed that Pink1 can regulate mitochondrial dynamics and morphology through the promotion of mitochondrial fission (Deng et al., 2008; Yang et al., 2008; Niu et al., 2019). Furthermore, liensinine, a newly identified mitophagy inhibitor that can exert synergistic effects with doxorubicin in the treatment of breast cancer, could inhibit doxorubicin-induced cardiotoxicity *via* the suppression of Drp1-mediated mitochondrial fission (Liang et al., 2020). In contrast, Wang et al. reported that mitophagy was activated and could suppress Drp1-induced mitochondrial fission in acute kidney injury (Wang et al., 2019). In terms of the mechanism, mitophagy could exert a protective effect against continuous, and harmful, mitochondrial fission. To a certain extent, this result was compatible with our findings that mitophagy may constitute a safeguard against the detrimental influence of mitochondrial fission. Combined, our findings demonstrated that mitochondrial fission and mitophagy exerted mutual promotive effects during CF activation, forming a mitochondrial fission–mitophagy positive feedback circuit that ensured continued CF activation. Meanwhile, this positive feedback mechanism could eliminate the detrimental influence of excessive mtROS generation resulting from mitochondrial fission, thereby helping to maintain intracellular homeostasis and CF survival.

Based on the important role of mitophagy in sustaining CF activation identified in the present study, this safeguarding mechanism for CF survival may aggravate cardiac fibrosis and heart failure. Although relatively few studies have investigated the role of mitophagy in the fibrotic heart, some have examined the effects of mitophagy in other fibrotic organs and reported results that may support the abovementioned view. Mitophagy-mediated self-renewal can accelerate the progression of lung and liver fibrosis and lead to organ failure (Larson-Casey et al., 2016; Qiu et al., 2019). However, other studies have demonstrated the essential role of mitophagy in maintaining normal cardiac function and protecting against acute cardiac injury (Campos et al., 2016; Bravo-San Pedro José et al., 2017; Luo et al., 2020). Under physiological conditions, mitophagy was shown to be essential for the normal perinatal transformation of myocardial metabolism (Gong et al., 2015). Following acute cardiac injury, such as myocardial infarction, mitophagy may also mediate robust cardioprotective effects. For example, the genetic deletion of Pink1 was reported to increase infarct size in response to ischemia–reperfusion injury (Siddall et al., 2013). Besides, parkin knockout can result in aggravated cardiac damage and reduced survival after ligation of the left anterior descending coronary artery in mice (Kubli et al., 2013). These harmful effects may be attributed to the antifibrotic effects associated with mitophagy deficiency, which resulted in delayed fibroblast-mediated repair and led to ventricular wall rupture in the acute phase of myocardial infarction. These sometimes contradictory results highlight the need for *in vivo* studies to elucidate the role of mitophagy in cardiac fibrosis. Considering that mitophagy may be critical for cardiomyocyte survival, it may restrict the *in vivo* application using non-specific siRNA-Pink1. Therefore, specific deletion of Pink1/Parkin in CF *via* mice expressing Cre recombinase linked to CF-specific promoter, Postn promoter, may be an ideal means in the future.

Our study had three main limitations. First, even though we validated the mitochondrial fission–mitophagy mutual reinforcement in activated CF, *in vivo* studies using animal models are needed to confirm our findings. Second, apart from the shift to glycolysis, we did not explore other profibrotic mechanisms associated with mitochondrial fission, such as cyclooxygenase-2 (COX-2)/prostaglandin E2 (PGE2)-dependent collagen production (Tseng et al., 2019). Third, although excessive mitophagy and defective mitochondrial biogenesis may be detrimental to cell survival, we did not explore the level of mitochondrial biogenesis during CF activation, which should be considered in the future.

Despite some limitations, we confirmed that enhanced mitochondrial fission can promote glycolysis during CF activation. Moreover, we identified a mitochondrial fission–mitophagy positive feedback circuit that helps to maintain CF activation and safeguard the health of activated CF.

## Data Availability Statement

The original contributions presented in the study are included in the article/Supplementary Materials, further inquiries can be directed to the corresponding author/s.

## Ethics Statement

The animal study was reviewed and approved by Institutional Animal Care and Use Committee, Sun Yat-sen University.

## Author Contributions

Y-XC, J-FW, and P-ML designed the study. Q-YG, H-FZ, JT, Z-TC, W-HL, and W-YY performed the *in vitro* experiments. Q-YG, H-FZ, M-XW, YX, C-YL, G-HG, and YY performed the statistical analyses and manuscript revision. Q-YG, H-FZ, and JT drafted the manuscript. Y-XC, J-FW, and P-ML helped to explain the critical points in the manuscript. All authors contributed to the article and approved the submitted version.

## Conflict of Interest

The authors declare that the research was conducted in the absence of any commercial or financial relationships that could be construed as a potential conflict of interest.
